The article "CD96 as a Potential Diagnostic Biomarker and New Target for Skin Cutaneous Melanoma" was published in 2022. Journal: Contrast Media Mol Imaging.

# CD96 as a Potential Diagnostic Biomarker and  New  Target for Skin Cutaneous Melanoma

**DOI:** 10.1155/2022/6409376

**Published:** 2022-08-08

**Authors:** Wangying Zhou, Xiaobin Cai, Feng Liu

**Affiliations:** Department of Plastic Surgery, Lishui Municipal Central Hospital, Affiliated Lishui Hospital of Zhejiang University, Zhejiang 323000, China

## Abstract

Skin cutaneous melanoma has high morbidity and mortality. Identification of reliable and quantitative melanoma biomarkers could facilitate an early diagnosis and improve survival and morbidity rates. CD96 has a significant role in adjusting immune function. Although the abnormal expression of CD96 has been reported to participate in carcinogenesis in many human types of cancer, the bioinformatics role of the CD96 in melanoma is unknown. Expression degrees and their underlying functions were first studied by this study. According to TCGA, GTEx, and gene expression profile interaction analysis dataset in this paper, compared with normal skin tissues, CD96 was expressed at higher levels in human cutaneous melanoma skin tissues. Meanwhile, we detected the relative CD96 expression levels by immunohistochemistry. Gene functional enrichment analyses were applied through cBioPortal database analysis. CD96 was clearly upregulated in skin cutaneous melanoma patients and carried out its effects through regulating several signaling pathways, containing the JAK-STAT, PI3K-Akt, and MAPK. Taken together, the analysis results indicated that CD96 could be used as a new clinical bioindicator as well as an underlying medicinal target for cutaneous melanoma.

## 1. Introduction

Melanoma is the deadliest skin malignity with a rising prevalence worldwide, of which the pathogenic mechanisms remain unclear as both environmental and genetic factors could contribute to its development [1] [2]. Even if apparent development has been made in surgical therapy, clinical diagnosis, and medical treatment covering immunotherapy and targeted treatment, patients have a very low 5-year survival rate [3]. Thus, it is urgent to investigate the initiation and developmental mechanisms in SKCM and to find novel combined molecular markers that may function as therapeutic targets for SKCM.

Cancer has been the number one killer gradually threatening our health in the past decades. New mechanisms and novel therapy for the treatment of cancer are constantly emerging. As we know, significant immunomodulatory effects are possessed by immune checkpoints. It was demonstrated that an effective strategy for treating cancer is to prohibit the immune checkpoint on the cell membrane [4]. CD96 belongs to the immunoglobulin superfamily [5]. cells and natural killer (NK) cells Its role in the regulation of immune function is crucial. Because of its underlying tumorigenicity and therapy, more and more oncology biologists recognize CD96. CD96 was demonstrated to restrain CD8+ T cells and NK cells which play an anticancer activity [6]. Tumor immunity was reported to be promoted by the lack of host CD96 and PD-1, but immune homeostasis was not significantly injured [7]. Several mouse tumor models were slowed by blocking CD96 [8]. Low expression of CD96 could reverse experimental lung cancer metastasis [8]. CD96 can be used as an oncogene, as the results suggested, and combined as a good therapeutic treatment target. What is not clear, however, is how CD96 in SKCM is associated with immune regulation and patient prognosis.

The article "CD96 as a Potential Diagnostic Biomarker and New Target for Skin Cutaneous Melanoma" was published in 2022. Journal: Contrast Media Mol Imaging.

As the high-throughput sequencing technologies develop [9], a key function in ascertaining biological and biomedical functions was shown by a large number of RNA and DNA studies [9]. The underlying function of CD96 in SKCM has not been explored by bioinformatics analysis, and potential biological functions of CD96 in SKCM were assessed.

## 2. Materials and Methods

### 2.1. CD96 Expression in Pan-Cancer

Users are permitted to conduct customized bioinformatics studies [10] with the relevant tools provided by the Sangerbox database (http://sangerbox.com/). Using Student's *t*-test, the gene CD96 expression levels in diverse specimens and corresponding normal controls were discussed according to the Cancer Genome Atlas (TCGA) and Genotype-Tissue Expression (GTEx) datasets. There was statistical significance when the *p* value was less than 0.05.

### 2.2. Gene Expression Profiling Interactive Analysis (GEPIA)

From TCGA and GTEx projects, RNA sequencing expression data were analyzed by this study from 8587 normal samples and 9736 tumor samples [11] using a latest developed interactive website—the online database Gene Expression Profiling Interaction Analysis (GEPIA) (http://gepia.cancer-pku.cn/). Differences in CD96 expression between SKCM and corresponding normal skin were detected. We conditioned the threshold on a *p* value of 0.01 and a multiplicative variation of 1, matching the GTEx data and TCGA normal data. In SKCM patients, by using the GEPIA dataset, the correlation between CD96 transcript levels and tumor stage was also measured and studied by us.

### 2.3. Immunohistochemistry Validation

From wide proteomic and transcriptomic information [12], we collected the mRNA expression patterns and proteins in tissues and cells in the Human Protein Atlas (HPA) (https://www.proteinatlas.org/), an extensive database [12]. As a result, the tissue and immune cell expression atlas of CD96 was analyzed by the HPA.

The article "CD96 as a Potential Diagnostic Biomarker and New Target for Skin Cutaneous Melanoma" was published in 2022. Journal: Contrast Media Mol Imaging.

Distinct CD96 expression in SKCM and normal skin tissues was verified by immunohistochemistry (IHC) according to the method described above [13]. Tissue slides were prepared following standard procedures, and rabbit polyclonal antibodies were used against CD96 (Abcam, ab264416) at 1/1000 dilution to incubate them at 4°C overnight. We next sliced them and combined them with horseradish peroxidase (HRP) antibody (1 : 200 dilution) for 2 hours at room temperature, then covered them with DAB (Vector Laboratories, Burlingame, CA), and we mounted slides with Vectashield mounting medium (Vector Laboratories). We used a Nikon E800 microscope to observe all sections.

### 2.4. cBioPortal Analysis

The cutaneous melanoma (TCGA, Firehose Legacy) dataset included 480 pathology-reported cases and was further studied for CD96 applying cBioPortal (https://www.cbioportal.org/) [14]. The mRNA expression z-scores (RNA Seq V2 RSEM), putative copy number alterations (CNA) of GISTIC, mutations, and protein expression z-scores (RPPA) were involved in the genomic alteration profile.

### 2.5. Protein-Protein Interaction (PPI) Network Construction

The PPI network was developed after the top 100 genes closely associated with CD96 alterations were entered into the STRING database (https://string-db.org/cgi/input.pl) [15], including physical and functional interactions. The cutoff of the PPI confidence score was set as 0.4.

### 2.6. Gene Ontology (GO) and Kyoto Encyclopedia of Genes and Genomes (KEGG) Pathway Analysis

R language software was employed, and enriched GO terms and signaling pathways of related genes closely associated with CD96 alterations were evaluated [16]. *p* value < 0.05 is the threshold of statistical significance for enrichment analysis, adjusted for *p* value < 0.05. This study showed the top 30 enriched pathways and top 10 GO terms for BP, CC, and MF.

## 3. Results

### 3.1. CD96 Expression Is Elevated in a Variety of Tumors

As shown in Figure 1(a), the CD96 expression level was significantly increased in a variety of tumors containing SKCM than that in the corresponding normal controls.

### 3.2. CD96 Is Upregulated in SKCM and Correlated with the Tumor Stage

CD96 expression level between SKCM and normal skin tissues was evaluated by GEPIA. As shown, CD96 expression level was significantly increased in SKCM compared with the normal skin tissue (Figure 1(b)). Tumor stage analysis also exhibited that CD96 expression levels were significantly different between groups in regard to tumor stage (Figure 1(c)).

CD96 proteins were expressed only in lung, salivary gland, spleen, lymph node, tonsil, and bone marrow tissues (Figure 2(a)).

The article "CD96 as a Potential Diagnostic Biomarker and New Target for Skin Cutaneous Melanoma" was published in 2022. Journal: Contrast Media Mol Imaging.

### 3.3. SKCM Patients

The CD96 alterations and neighbor genes correlated with CD96 alterations were analyzed in SKCM by cBioPortal database. As shown, CD96 alteration included deep deletion, mRNA upregulation, splice mutation, and missense mutation (Figures 3(a) and 3(b)). The whole altered neighbor genes correlated with CD96 were listed. The results showed that P2RY10, LCK, SLAMF6, IKZF1, CD2, CD247, TIGIT, TRAT1, CD3G, SLA2, and so on were closely associated with CD96 alterations in SKCM (Table 1). Meanwhile, Figure 3(c) shows the involvement and association among the genes in PPI network.

### 3.4. GO and KEGG Enrichment Analysis

Figure 4 shows post-translational protein modification, RNA catabolic process, etc. The genes in the CC terms were strongly enriched in focal adhesion, cell-cell junction, cell-substrate junction, etc.

For KEGG pathway visualization, we found that apoptosis and proliferation of cells were significantly more apoptotic in related pathways (Figure 5). Nevertheless, the most significant enrichment signaling pathway included multiple inflammatory-related signaling pathways (Figure 5). Also, tumor-related signaling pathways containing gastric cancer and breast cancer were significantly enriched.

## 4. Discussion

Although the function of CD96 in the pan-cancer pattern has been partly explored, further demonstration of a certain relationship between CD96 and cancers is very important. Our study provided a novel idea to explore the correlation between CD96 expression and SKCM.

In the study, we found that CD96 was upregulated in various types of cancers from the data in TCGA and GTEx dataset (Figure 1(a)). GEPIA databases manifested that the expression of CD96 was higher in SKCM samples than that of normal skin tissues (Figure 1(b)), and it was significantly correlated with the tumor stage (Figure 1(c)). Furthermore, IHC also exhibited that CD96 expression was upregulated in SKCM tissues (Figure 2). Moreover, CD96 alterations were analyzed by cBioPortal, and joint analysis was performed by PPI and GO and KEGG enrichment. As shown in Figure 4, clinically important module genes of SKCM in the GO analysis contained RNA catabolic process, focal adhesion, cell-cell junction, cell-substrate junction, cadherin binding, ATPase activity, etc. (Figure 5). The results of our analysis prove that CD96 may be a powerful biomarker for SKCM diagnosis and drug discovery.

## 5. Conclusion

In conclusion, our study demonstrated a higher expression level of CD96 in cutaneous skin melanoma. Abnormally expressed CD96 was significantly related to the stage of skin cutaneous melanoma. Moreover, CD96 alterations were closely related with multiple cell functions such as post-translational protein modification, cell-cell junction, cadherin binding, and so on. Additionally, cell apoptosis and proliferation and inflammatory-related and cancer-related signaling pathways were significantly enriched through the gene with CD96 alterations. This study provides a new idea for using the public genome information databases to excavate and obtain specific gene information for certain cancer. Our findings showed that CD96 may serve as a new gene for the diagnosis and treatment of skin cutaneous melanoma patients. However, these results need to be verified by large-scale clinical investigations and verification experiments in vitro and in vivo.

The article "CD96 as a Potential Diagnostic Biomarker and New Target for Skin Cutaneous Melanoma" was published in 2022. Journal: Contrast Media Mol Imaging.

## Figures and Tables

**Figure 1:** CD96 was upregulated in skin cutaneous melanoma. (a) The expression level of CD96 was increased in multiple types of tumors compared with normal samples. (b) The expression level of CD96 was increased in skin cutaneous melanoma compared with normal skin samples. (c) Significant relationship was found in skin cutaneous melanoma tumor stage with CD96 expression level by GEPIA (^*∗*^*p* < 0.05, ^*∗∗*^*p* < 0.01, and ^*∗∗∗*^*p* < 0.001).

**Figure 2:** Expression level of CD96. (a) CD96 protein expression. (b) CD96 mRNA expression level. (c) CD96 mRNA expression level in different immune cells. (d) CD96 protein expression in skin cutaneous melanoma and corresponding normal skin tissue detected by IHC.

**Figure 3:** CD96 gene mutation analysis in skin cutaneous melanoma. (a, b) Acquiring mutation information of CD96 using cBioPortal. (c) PPI network of the top 100 correlated genes.

**Figure 4:** GO enrichment analysis of CD96 and genes correlated with CD96 alterations by R language software.

**Figure 5:** KEGG enrichment analysis of CD96 and genes correlated with CD96 alterations by R language software.

**Table 1:** Genes are correlated with CD96 in skin cutaneous melanoma.

Correlated gene	Cytoband	Spearman's correlation	*p* value	*q* value
P2RY10	Xq21.1	0.917792370177848	1.16269632845918*E* − 190	2.32818312810666*E* − 186
LCK	1p35.2	0.914186998262427	1.8019658692741*E* − 186	1.80412822831723*E* − 182
SLAMF6	1q23.2-q23.3	0.913079755637399	3.20377136123396*E* − 185	2.13841059124496*E* − 181
IKZF1	7p12.2	0.9108928449566	8.43332045425359*E* − 183	4.22172021939934*E* − 179
CD2	1p13.1	0.910340509960402	3.36839457860001*E* − 182	1.34897466083773*E* − 178
CD247	1q24.2	0.907572698456952	3.0458209366593*E* − 179	8.87185028600711*E* − 176
TIGIT	3q13.31	0.907565223675281	3.10142588903564*E* − 179	8.87185028600711*E* − 176
TRAT1	3q13.13	0.906742618574921	2.2499382652113*E* − 178	5.63159547782389*E* − 175
CD3G	11q23.3	0.906349373592915	5.76451363930558*E* − 178	1.28254023459394*E* − 174
SLA2	20q11.23	0.905792901587852	2.16707171454158*E* − 177	4.33934440119807*E* − 174

The article "CD96 as a Potential Diagnostic Biomarker and New Target for Skin Cutaneous Melanoma" was published in 2022. Journal: Contrast Media Mol Imaging.

## Data Availability

The experimental data used to support the findings of this study are available from the corresponding author upon request.
